# Usefulness of Continuous Low-Dose Fentanyl in Combination with Dexmedetomidine and Midazolam for Intravenous Sedation: A Randomised Controlled Trial

**DOI:** 10.1155/2022/2807581

**Published:** 2022-05-16

**Authors:** Yoko Okumura, Aiji Sato (Boku), Naoko Tachi, Mayuko Kanazawa, Miko Kawabata, Masahiro Okuda

**Affiliations:** Department of Anesthesiology, School of Dentistry, Aichi Gakuin University, 2-11 Suemori-Dori, Nagoya, Aichi 464-8651, Japan

## Abstract

Intravenous dexmedetomidine (DEX) and midazolam (MZ) are currently used to achieve sedation in dental surgery under local anaesthesia. However, the efficacy of low-dose fentanyl (FEN) in combination with DEX and MZ sedation remains unclear. Therefore, we implemented a prospective randomised controlled trial to investigate the intra- and postoperative analgesic effects, intraoperative respiratory and circulatory dynamics, and frequency of intra- and postoperative adverse events of continuous low-dose fentanyl administration with DEX and MZ sedation. Patients aged 20–64 years scheduled for dental surgery under sedation were randomly assigned to the DEX+MZ (DM) or DEX+MZ+FEN (DMF) group. DEX was administered at 4 *μ*g/kg/h for 10 min and then reduced to 0.7 *μ*g/kg/h until the end of surgery. MZ was administered at 0.04 mg/kg upon the initial administration of DEX and 0.02 mg/kg every hour thereafter. In the DMF group, FEN infusion was administered at 2 *μ*g/kg/h during the initial administration of DEX and then reduced to 1 *μ*g/kg/h after 10 min until the end of surgery. Primary outcomes were intra- and postoperative analgesic efficacies, whereas secondary outcomes were intraoperative respiratory and circulatory dynamics. The total amount of intraoperative local anaesthetic administered and the heart rate were significantly lower in the DMF group than in the DM group (*P* = 0.044 and *P* < 0.01, respectively). No significant difference was observed in the frequency of postoperative administration of analgesics and intra- and postoperative adverse events. These findings demonstrated that low-dose FEN infusion in combination with DEX and MZ sedation in dental surgery provides intraoperative analgesia and suppresses tachycardia with little effect on blood pressure and respiratory dynamics and without effect on postoperative analgesia.

## 1. Introduction

Intravenous sedation for dental surgery is provided to reduce patients' anxiety and nervousness, enabling patient cooperation with the surgical procedure and controlling their body movement for safer surgery. In general, both the patient and dental surgeon desire intraoperative amnesia and quick postoperative recovery; therefore, midazolam (MZ) and/or propofol is often administered as sedatives given their amnesic effects. However, pharyngeal reflex suppression and respiratory depression, which may occur as the level of consciousness decreases, have raised concerns related to the occurrence of aspiration and airway obstruction upon water injection during dental surgery.

Dexmedetomidine (DEX) has recently become a popular intravenous sedative in dental surgery under local anaesthesia [1]. It is an agonist of *α*-2A-adrenergic receptors in the locus ceruleus with sedative effects mirroring that of physiologic sleep. Therefore, patients under DEX sedation can be easily roused with a call and do not develop respiratory suppression even at high doses [2]. These pharmacologic characteristics are useful in avoiding aspiration and airway obstruction during dental surgery. However, given that DEX does not have an amnesic effect, patients may retain the memory of the surgery upon awakening from the sound or vibration of cutting instruments, treatment-associated pain, and name-calling. Consequently, DEX is usually administered with a small amount of MZ during dental surgery. Moreover, opioid analgesics may be used as an adjunct during intravenous sedation for dental surgery [3]. We have previously shown that intravenous sedation with propofol plus continuous low-dose fentanyl (FEN) stabilised intraoperative respiratory and circulatory dynamics and reduced postoperative pain [4]. However, the sedative, amnesic, and analgesic effects and safety of combining DEX and MZ sedation with continuous low-dose FEN remain unclear.

The current study was aimed at investigating the intra- and postoperative analgesic effects, intraoperative respiratory and circulatory dynamics, and frequency of intra- and postoperative adverse events of continuous low-dose FEN in combination with conventional intravenous sedation with DEX and MZ. We hypothesised that the addition of continuous low-dose FEN to sedation using DEX and MZ was associated with more effective intra- and postoperative analgesia and reduced respiratory and circulatory depression compared with that of DEX and MZ sedation alone.

## 2. Materials and Methods

### 2.1. Ethics Approval and Consent to Participate

This study was performed following the ethical standards of the Declaration of Helsinki (1964) and its subsequent amendments. This study adhered to the Consolidated Standards of Reporting Trials guidelines; was approved by the ethics committee of the School of Dentistry, Aichi Gakuin University, on 9 November 2018 (Approval No. 544); and was registered in the UMIN-ICDR on 20 November 2018 (UMIN study ID: UMIN000034929) before the start of the clinical study. The first patient was recruited and registered on 21 November 2018. After providing sufficient explanation to all patients, written informed consent was obtained before study participation.

### 2.2. Study Design and Population

This prospective randomised controlled study enrolled 85 patients aged 20–64 years who were scheduled for dental surgery that was expected to last for more than 1 hour. All patients were classified as American Society of Anesthesiologists physical status class 1 or 2 and received sedation with either DEX+MZ (DM) or DEX+MZ+FEN (DMF) groups. Patients with uncontrolled hypertension (*n* = 1) and hyperthyroidism (*n* = 1), those who were obese (body mass index of ≥30; *n* = 7), and those who did not provide consent (*n* = 3) were excluded. Overall, the final study population comprised 73 patients who were randomly divided into the DM (*n* = 31) and DMF groups (*n* = 42). A researcher who was not in charge of providing anaesthesia conducted the randomisation using computer-generated random numbers (Figure 1).

### 2.3. Anaesthesia Methods

Anaesthesia management was performed by several dental anaesthetists who had at least 3 years of experience in intravenous sedation for dental surgery. The surgery was performed by two surgeons with at least 3 years of experience in dental surgery. Patients were instructed to fast after midnight on the day of the surgery and were allowed to drink clear water until 2 h preoperatively. Patients were not administered any preanaesthetic medication. Each patient was placed in a supine position on the operating table, followed by the attachment of an electrocardiograph, blood pressure metre, pulse oximetre, and nasal cannula with an expiratory gas sampling tube for oxygen delivery at 2 L/min, which measures _ET_CO_2_ and respiratory rate. Subsequently, the venous route was secured in the left or right forearm. Appropriate DEX, MZ, and FEN doses were calculated to target the predicted intraoperative effect-site concentrations, as previously reported by Dyck et al., Zomorodi et al. and Shafer et al [5–7] using the AnestAssist® [8] before entering the operating room.

DEX was administered at 4 *μ*g/kg/h to maintain an intraoperative effect-site concentration of approximately 0.6 ng/mL for appropriate sedation [5] and was reduced to 0.7 *μ*g/kg/h 10 min after the induction of anaesthesia until the end of surgery. MZ was administered at 0.04 mg/kg upon starting DEX and at 0.02 mg/kg every hour thereafter to maintain an intraoperative effect-site concentration of approximately 75 ng/mL, which was expected to have an amnesic effect [6]. In the DMF group, continuous FEN infusion was started 2 *μ*g/kg/h upon starting DEX administration and reduced to 1 *μ*g/kg/h 10 min after the induction of anaesthesia until the end of surgery to target a predicted intraoperative effect-site concentration of 0.6 ng/mL for mild analgesia [7, 9].

The intraoperative bispectral index (BIS) value was maintained within 70–80 based on the reported anaesthetic management by Tagawa et al. [10]. When the BIS value was increased to >85, along with an OAA/S score of ≥4, 0.02 mg/kg of MZ was administered as a bolus dose. If no spontaneous breathing occurred and the peripheral oxygen saturation (SpO_2_) was <89%, the anaesthetist provided verbal instructions for the patient to breathe. If patients could not follow verbal instructions, mandibular elevation was performed. When the anaesthetist determined that the analgesia was inadequate based on patients' complaints and body movements, the anaesthetist asked the surgeon to properly administer a local anaesthetic using ORA® Injection Dental Cartridge, a dental cartridge formulation of 2% lidocaine containing 1/72,780 adrenaline. Immediately before the end of the surgery, 50 mg of flurbiprofen axetil or 1000 mg of acetaminophen was administered intravenously (Figure 2).

A total of 50 patients were randomly allocated to treatment with dexmedetomidine (DEX) and midazolam (MZ) (DM group) or treatment with continuous infusion of low-dose fentanyl (FEN) combined with DEX and MZ (DMF group). During treatment, an additional 0.02 mg/kg of MZ was administered every 60 min. If the patient was not adequately sedated, a single intravenous bolus of MZ 0.02 mg/kg was given to achieve a bispectral index (BIS) value of approximately 70–80.

### 2.4. Measurements

The primary outcomes were intra- and postoperative analgesic efficacy, including the dose of local anaesthetics, the time elapsed from the time of leaving the operating room to the first analgesic administration, and the number of analgesic doses needed from the time the patient left the operating room until 9:00 AM of the next day. Secondary outcomes were intraoperative respiratory and circulatory dynamics, including the respiratory rate, SpO_2_, P_ET_CO_2_, heart rate, and mean blood pressure. Other variables investigated were DEX, MZ, and FEN doses and the number of additional MZ doses needed to maintain BIS at 70–80, intraoperative memory, and the frequency and types of adverse events. These were extracted from a database recorded by PaperChart® [11], an automated anaesthesia recording software.

### 2.5. Statistical Analysis

Based on the set effect size of 1.0, minimal significance (*α*) of 0.05, and statistical power (1 − *β*) of 0.95, the minimum sample number was estimated to be 46 patients (*n* = 23 per group). The effect size was calculated based on the statistical analysis results of a pilot study that used intra- and postoperative analgesic efficacy as the standard anaesthesia (DM group, *n* = 10, and DMF group, *n* = 10). Given that the use of statistical tests in the absence of a reliable calculation decreases the weight of the sample size, our final sample size was calculated considering an expected dropout rate of 0.05 based on our pilot study. Therefore, if a dropout rate (*R*) is expected, a simple but adequate adjustment is provided using *N*_*d*_ = *N*/(1 − *R*)^2^, where *N* is the calculated sample size assuming no dropout and *N*_*d*_ is the estimated sample size required when dropouts are expected [12, 13]. Therefore, after adjusting for dropouts, a final sample of 50 patients was estimated.

Differences in age, height, weight, operative time, anaesthesia time, and the total amount of administered DEX, which were determined to have a normal distribution on normality testing, were analysed using Student's *t*-test. Differences in the total amount of administered local anaesthetics and MZ and the duration between leaving the operating room and the first analgesic administration, which were determined to have a nonnormal distribution on normality testing, were analysed using Welch's *t*-test. Differences in the number of required additional MZ doses were analysed using the Mann–Whitney *U* test. Differences in sex, operative procedure, underlying disease, number of analgesic doses needed after leaving the operating room until 9:00 AM of the next day, and the frequency of intra- and postoperative adverse events were compared using the *χ*^2^ test. Multiple measurements of intraoperative respiratory and circulatory dynamics were compared using a two-way analysis of variance. Statistical significance was set at a *P* value of <0.05.

## 3. Results

### 3.1. Patient Characteristics

No significant differences in age, height, weight, sex, underlying disease, operative time, anaesthesia time, and surgical technique were observed between the two groups (Table 1).

### 3.2. Intra- and Postoperative Analgesic Efficacy

The total amount and the number of administered local anaesthetic dose were significantly lower in the DMF group than in the DM group (*P* = 0.044 vs. 0.038, respectively) (Table 2). Regarding the postoperative analgesic efficacy, no significant differences were observed in the time elapsed after leaving the operating room until the first administration of analgesic, and the number of analgesic doses needed after leaving the operating room until 9:00 AM of the next day postoperatively were observed between the two groups (Table 3).

### 3.3. Sedative Effect

We then compared the total amounts of DEX, MZ, and FEN and the number of additional MZ doses needed to maintain BIS values within 70–80 between the two groups. Accordingly, no significant differences in the total amounts of DEX and MZ were observed between the two groups (Table 4). Similarly, based on the discretion of shallow sedation level by the anaesthetists, no significant difference in the number of patients who needed additional MZ doses was observed between the DM (*n* = 14) and DMF (*n* = 13) groups. Moreover, the total amount of administered MZ was similar between the two groups (Table 4).

### 3.4. Respiratory and Circulatory Dynamics

Regarding the intraoperative respiratory dynamics (Figure 3), no significant differences in the respiratory rate (Figure 3(a)), SpO_2_ (Figure 3(b)), and P_ET_CO_2_ (Figure 3(c)) were observed between the two groups. One patient in the DM group needed mandibular elevation for respiratory support. Regarding the intraoperative circulatory dynamics (Figure 4), both groups had similar mean arterial pressure (Figure 4(a)), whereas the DMF group had a significantly lower heart rate (Figure 4(b)) than the DM group (*P* < 0.01). No patient in either group was administered circulatory agonists.

### 3.5. Frequency and Details of Intra- and Postoperative Adverse Events

Intraoperative adverse events detected included body movements, the need for mandibular elevation, and gastric juice vomiting. In the DM group, mandibular elevation was needed for one patient, body movements were observed in two patients, and gastric juice vomiting was observed in one patient intraoperatively (Table 5). Aspiration and accidental ingestion were prevented by turning the patient's head to the left and by immediately suctioning the gastric juice by the surgeon. Meanwhile, no adverse events were mentioned in the anaesthesia records of patients in the DMF group. No significant differences in the frequency of intraoperative adverse events were observed between the two groups.

Nausea and/or vomiting occurred in two patients in the DM group and four in the DMF group postoperatively (Table 6). The systolic blood pressure dropped to <80 mmHg in three and one patient in the DM and DMF groups, respectively. For these patients, passive leg raising and increased intravenous fluid administration rate were performed. None of them received vasopressor agents. Five patients in each group had residual intraoperative memory. No significant differences in the frequencies of postoperative adverse events were observed between the two groups.

## 4. Discussion

In the current study, continuous infusion of low-dose FEN in combination with DEX and MZ sedation in dental surgery reduced the amount of local anaesthetic used. Local dental anaesthetics was administered by the surgeon according to the request of the anaesthetist. This was done after the anaesthetist had determined that the amount of analgesia administered to the patient was inadequate based on the patient's complaints and body movements during the surgical procedure. Based on the significantly lower amount of administered local anaesthetic in the DMF (5.4 mL) than in the DM group (7.2 mL), low-dose FEN may enhance the intraoperative analgesic effect during dental surgery under DEX and MZ sedation. Conversely, the two groups had no significant difference in terms of the total amount of postoperative analgesics and the time elapsed after leaving the operating room until the first analgesic administration. Therefore, intraoperative administration of low-dose FEN did not influence postoperative analgesia.

Local dental anaesthetic cartridges were supplemented with adrenaline at a concentration of approximately 1/80,000 to prolong the duration of action. Furthermore, this step increased cardiac output in a dose-dependent manner, thereby increasing the heart rate and cardiac contractility. Therefore, the Japanese Dental Society of Anesthesiology had explained in its “Statement on Safe Local Dental Anaesthesia” that 3–5 mL of the anaesthetic should be used as a dental surgery guideline, which should be increased or decreased based on age, anaesthetic area, site, tissue, symptoms, and histology while considering the standard maximum dose of adrenaline [14]. Furthermore, the same society has recommended that the local anaesthetic dosage should be limited to 3.6 mL for patients with hypertension and be discontinued if the systolic and diastolic blood pressures exceeds 180 mmHg and 90 mmHg, respectively [15]. In the current study, the heart rate was significantly lower in the DMF group than in the DM group; thus, low-dose FEN in combination with DEX and MZ intravenous sedation may be useful for hemodynamic stability during dental surgery by suppressing tachycardia without causing unstable hypotension or bradycardia for healthy adult patients.

The respiratory depressant effect of DEX is minimal when administered alone [7] but increases when administered with MZ and/or FEN. In the current study, although one patient in the DM who did not receive FEN needed mandibular elevation because of unresponsiveness and SpO_2_ of <89% intraoperatively, both groups had similar respiratory rates, SpO_2_, P_ET_CO_2_, and total amount of MZ. Therefore, low-dose FEN did not exacerbate the respiratory depressant effect of DEX and MZ sedation. Furthermore, some patients in the DM group experienced body movements and gastric juice vomiting. Although intraoperative adverse events did not occur in the DMF group, the intergroup frequency was similar. The postoperative adverse events included nausea and/or vomiting (PONV; DM group *n* = 2, DMF group *n* = 4), hypotension (DM group *n* = 4, DMF group *n* = 1), and residual intraoperative memory (DM group *n* = 5, DMF group *n* = 5). None of these patients received antiemetic or antihypertensive drugs. Owing to the fact that bradycardia was not observed in any of the patients, the hypotension was mainly attributed to the *α*2 action of DEX [16]. Furthermore, the frequency of postoperative adverse events was similar between the two groups. Based on our results, low-dose FEN in combination with DEX and MZ intravenous sedation did not increase the frequency of intra- and postoperative adverse events.

Wang et al. [1] reported that, in dental implant placement, DEX reduced the intraoperative heart rate significantly more than MZ and had a lower VAS pain score 135 minutes after the start of anaesthetic administration. Furthermore, in the DEX group of Wang et al. [1], the time from the start of anaesthetic administration until the use of analgesics was approximately 4 hours. In the current study, flurbiprofen axetil or acetaminophen was used at the end of surgery, and the time from the start of anaesthetic administration to the use of analgesics (as in Wang et al. [1]) was approximately 6 hours in both the DM and DMF groups. Therefore, although intraoperative low-dose fentanyl did not have a postoperative analgesic effect, the intraoperative use of nonsteroidal anti-inflammatory analgesics may have prolonged the postoperative analgesic effect of DEX.

Togawa et al. [10] reported significantly fewer cases of intraoperative body movement with DEX and MZ sedation than with P and MZ sedation. In the current study, intraoperative adverse events were extracted from the anaesthesia records, indicating that adverse events such as body movements were regarded as relatively severe by the anaesthesiologist. Consequently, a patient movement score 2 was seen in 3 patients (7%) in the DM group of Togawa et al. [10], and we saw this in 2 patients (8%) in the DM group and 0 patients (0%) in the DMF group in the present study. Moreover, Togawa et al. [10] reported one case (2%) in which it was impossible to control body movements. In the current study, one case (4%) who underwent wisdom tooth extraction under DM anaesthesia was excluded because hyperventilation which arose by insertion of the elevator immediately after the start of the surgery could not be controlled. DEX administration was discontinued based on previous successful outpatient clinic experiences on intravenous sedation with propofol alone for multiple dental treatments in patients with dental phobia. However, in the aforementioned case, hyperventilation was not completely controlled even with propofol. Dental phobia was not an exclusion criterion in this study given that DEX had been reportedly useful for sedation in such cases [17, 18]. However, a reexamination of the anaesthesia records to determine reasons for DEX discontinuation postoperatively revealed that the time of local anaesthesia infiltration and the start of surgery coincided. Considering that the surgery had been started before achieving local anaesthesia, hyperventilation may have been caused by pain as an awakening stimulus, which may be reduced with fentanyl. The DM and DMF groups of the present study had a slightly higher number of patients who had no intraoperative memory than the DM group of Togawa et al. (80% vs. 68%) [10]. This may be due to the use of double doses of MZ at induction of anaesthesia in the present study. Other postoperative complications were similar to those in the current study.

This study has several limitations. First, patients under sedation cannot be properly assessed using the VAS pain score. Therefore, in this study, anaesthesiologists with at least 3 years of experience in the anaesthetic management of intravenous sedation made judgements based on patient statements and body movements. Second, obese patients and the elderly would overdose if benzodiazepines and opioids were administered as in this study, leading to respiratory and circulatory depression. Third, poorly controlled hypertension and hyperthyroidism were risk factors for the development of abnormal hypertension and hypotension due to DEX, and thus, we excluded these patients from the study. Fourth, because patients under DEX sedation are aroused by stimulation, severely dental-phobic patients may not be able to maintain sedation when aroused by significant pain stimulation. Further investigation is needed to determine whether low-dose fentanyl is useful for such patients.

## 5. Conclusions

Continuous infusion of low-dose FEN in combination with DEX and MZ sedation in dental surgery provides intraoperative analgesic effects given its ability to reduce the amount of local anaesthetic used, as well as suppress tachycardia, with little effect on blood pressure and respiratory dynamics intraoperatively, while not affecting the postoperative analgesic effect.

## Figures and Tables

**Figure 1:** Consolidated Standards of Reporting Trials flow diagram.

**Figure 2:** Study protocol for the randomised controlled study.

**Figure 3:** Intraoperative respiratory dynamics: (a) respiratory rate; (b) SpO_2_; (c) P_ET_CO_2_. Values represent mean ± standard deviation. Abbreviations: SpO_2_: oxygen saturation; P_ET_CO_2_: end-tidal CO_2_.

**Figure 4:** Intraoperative circulatory dynamics: (a) mean arterial pressure; (b) heart rate. Values represent mean ± standard deviation. ^∗∗^*P* < 0.01 versus group DM.

**Table 1:** Patient characteristics. Values represent mean ± standard deviation.

	Group DM (*n* = 25)	Group DMF (*n* = 25)	*P*
Age (years)	40.6 ± 14.8	36.4 ± 12.1	0.377
Height (cm)	160.5 ± 8.0	164 ± 8.4	0.273
Weight (kg)	56.6 ± 9.7	58.5 ± 12.0	0.536
Sex (male : female)	5 : 20	12 : 13	0.090
Underlying disease			
Hypertension and diabetes mellitus	1	0	
Hypertension	0	1	
Depression	1	0	
Epilepsy	0	1	
None	23	23	1.000
Operation time (min)	64.1 ± 24.9	54.3 ± 21.4	0.144
Anaesthesia time (min)	77.4 ± 24.4	87.3 ± 27.0	0.181
Operative procedure	25	25	0.938
Extraction of impacted wisdom teeth	7	6	
Root-canal cystectomy	3	4	
General teeth extraction	3	4	
Dental implant placement	4	3	
Alveoloplasty	2	1	
Removal of metal plates in the maxilla and mandible	3	4	
Others	3	3	

**Table 2:** Intraoperative analgesic efficacy represented as differences in the local anaesthetic dosage and the number of additional local anaesthetic doses. ^∗^*P* < 0.05 versus DM group.

	Group DM (*n* = 25)	Group DMF (*n* = 25)	*P*
Total amount of local anaesthetic (mL) median (1st–3rd quartile)	7.2 (4.5–9.0)	5.4 (3.6–7.2)	0.044^∗^
Number of additional local anaesthetic dose (*n*) median (1st−3rd quartile)	1 (0–2)	0 (0–1)	0.038^∗^

**Table 3:** Postoperative analgesic efficacy represented as differences in the time elapsed after leaving the operating room until the first analgesic administration and the number of analgesic doses needed after leaving the operating room until 9:00 AM of the next day.

	Group DM (*n* = 25)	Group DMF (*n* = 25)	*P*
Time elapsed after leaving the operating room until the first analgesic administration (min) (mean ± SD)	287.8 ± 169.7	306.6 ± 164.1	0.734
Number of analgesic doses needed after leaving the operating room until 9:00 AM of the next day (mean ± SD)	1 (0–2)	1 (0–2)	0.691

**Table 4:** Total amounts of dexmedetomidine, midazolam, and fentanyl and the number of additional midazolam doses.

	Group DM (*n* = 25)	Group DMF (*n* = 25)	*P*
Total amount of DEX (*μ*g) (mean ± SD)	86.5 ± 16.7	84.8 ± 24.3	0.794
Total amount of FEN (*μ*g) median (1st−3rd quartile)	0	85 (50–15)	—
Total amount of MZ (mg) median (1st−3rd quartile)	4 (3–4.5)	4 (3.5–5)	0.388
Number of additional MZ dose (*n*) median (1st−3rd quartile)	1 (0–2)	1 (0–1)	0.614

**Table 5:** Frequency and details of intraoperative adverse events.

	Group DM (*n*)	Group DMF (*n*)	*P*
Frequency of intraoperative adverse events	5	0	0.226
Body movements	2	0	—
Performed mandibular elevation	1	0	—
Gastric juice vomiting	1	0	—
None	21	25	—

**Table 6:** Frequency and details of post–operative adverse events.

	Group DM (*n*)	Group DMF (*n*)	*P*
Frequency of post–operative adverse events	10	10	0.644
Nausea and/or vomiting	2	4	—
Systolic blood pressure < 80 mmHg	3	1	—
Residual intra–operative memory	5	5	—
None	15	15	—

## Data Availability

The data presented herein are not publicly available due to a lack of previous approval by the Research Ethics Committee but are available on request from the corresponding author.
